The article "MicroRNA profiling in gingival crevicular fluid of periodontitis—a pilot study" was published in 2017. Journal: FEBS Open Bio.

# MicroRNA profiling in gingival crevicular fluid of periodontitis—a pilot study

**DOI:** 10.1002/2211-5463.12238

**Published:** 2017-06-05

**Authors:** Akira Saito, Masafumi Horie, Kenichiro Ejiri, Akira Aoki, Sayaka Katagiri, Shogo Maekawa, Shinta Suzuki, Sophannary Kong, Tsuneto Yamauchi, Yoko Yamaguchi, Yuichi Izumi, Mitsuhiro Ohshima

**Affiliations:** ^1^ Department of Respiratory MedicineGraduate School of MedicineThe University of TokyoJapan; ^2^ Division for Health Service PromotionThe University of TokyoJapan; ^3^ Division of Genomic Technologies (DGT)RIKEN Center for Life Science TechnologiesYokohamaKanagawaJapan; ^4^ Department of PeriodontologyGraduate School of Medical and Dental SciencesTokyo Medical and Dental University (TMDU)Japan; ^5^ Department of MathematicsKeio UniversityYokohamaKanagawaJapan; ^6^ Department of BiochemistryNihon University School of DentistryTokyoJapan; ^7^ Department of BiochemistryOhu University School of Pharmaceutical SciencesKoriyamaFukushimaJapan

**Keywords:** gingival crevicular fluid, microRNA, periodontal pocket, periodontitis

## Abstract

Periodontitis is a chronic inflammatory disease that affects the interface of teeth and surrounding tissues. Gingival crevicular fluid (GCF) is an exudate of the periodontal tissues and can be collected from the gap between the tooth and gum (gingival sulcus or periodontal pocket) with paper strips. Testing of GCF is a low‐cost and minimally invasive procedure. In a variety of diseases, microRNAs (miRNAs) in body fluids are implicated in pathogenesis, and are suggested as potential diagnostic biomarkers. Here, we profiled miRNAs in GCF (two chronic periodontitis, one aggressive periodontitis, and five healthy subjects) using miRCURY LNA™ Universal RT microRNA PCR System, which yielded quantitative measures of more than 600 miRNAs. Through this analysis, we found that miRNA profiles in GCF of periodontitis patients are distinct from those of healthy controls. We further selected 40 miRNAs and confirmed their differential expression patterns in different subjects (five chronic periodontitis, one aggressive periodontitis, and six healthy subjects) using a custom miRNA PCR panel. This is the first demonstration of miRNA profiling in GCF and its alteration in periodontitis. Our findings suggest that a subset of miRNAs in GCF holds potential as a biomarker for periodontitis.

**Abbreviations**
BOP: bleeding on probing
Cq: quantitation cycle
ECM: extracellular matrix
FDR: false discovery rate
GCF: gingival crevicular fluid
PCA: principal component analysis
PD: periodontal pocket depth
VEGF: vascular endothelial growth factor

Periodontitis is one of the most common diseases and its prevalence has been estimated as almost half of the adult population in the United States 1. Periodontitis is a chronic inflammatory disease that affects the interface of tooth and periodontal tissues such as gingiva, root cementum, periodontal ligament, and alveolar bone. In advanced periodontitis, deepening of periodontal pockets, loss of tooth‐supporting connective tissues' attachment as well as alveolar bone resorption occur, eventually leading to tooth mobility and tooth loss. The associations between periodontitis and other common systemic diseases have been demonstrated, such as metabolic syndrome 2, coronary artery disease 3, and diabetes mellitus 4. These observations imply that prevention and treatment of periodontitis is of clinical importance in terms of maintaining good general health condition.

Currently, the diagnosis and classification of periodontitis mainly rely on conventional clinical assessments such as measurement of pocket depth (probing), dental plaque accumulation, bleeding on probing (BOP), and radiographic examination of alveolar bone loss. The evaluation of these clinical parameters except for radiography is largely dependent on the experience and skills of the dentists, and there could be disagreement in clinical judgment. Thus, alternative diagnostic methods based on objective and quantitative measures are in need to assist the diagnosis of periodontitis.

Gingival crevicular fluid (GCF) is an exudate of the periodontal tissues and is collected with paper strips. The collection of GCF can be performed easily and quickly with a minimally invasive procedure. GCF samples contain a variety of proteins and nucleic acids, providing useful information for the diagnosis of periodontal diseases 5. We have previously demonstrated that the levels of growth factors and cytokines are indicative of periodontal disease activity 6, 7, 8. These findings support the notion that detection of biomarkers in GCF holds potential to improve the diagnostic accuracy of periodontitis. Furthermore, the advantage of testing GCF rather than saliva is that the information of individual periodontal site is directly linked to the diagnosis for each tooth.

MicroRNAs represent a group of short noncoding RNAs that regulate expression of proteins by binding to the 3′UTRs of target mRNAs. In mammalian cells, the primary transcripts of miRNAs (pri‐miRNAs) are transcribed from miRNA‐coding sequences. Most pri‐miRNAs are processed into short hairpin RNAs (precursor miRNAs) by the Drosha/DGCR8 complex and are further cleaved by Dicer to yield miRNA duplexes of 21–25 nucleotides in length. The mature miRNA strand is subsequently incorporated into the RNA‐induced silencing complex (RISC) that is directed to complementary mRNAs for gene silencing 9. Many miRNA families are evolutionarily conserved and the latest release of mirbase (version 21) includes 1881 precursor and 2588 mature miRNAs in humans 10.

Gene regulation by miRNAs is vital in a variety of biological or pathological processes, such as pluripotency 11, cell differentiation 12, and carcinogenesis 13. Accumulating evidence suggests that every kind of body fluid contains miRNAs that reflect the disease status and they act as diagnostic biomarkers. Indeed, increasing efforts are made for the development of cancer diagnostic tools that detect miRNAs in blood, urine or other body fluids 14. However, the roles of miRNAs in periodontal diseases have been fragmentarily described and it remains unknown whether GCF contains miRNAs, and if this is the case, specific miRNAs are diagnostic for periodontitis.

We postulated that GCF might contain miRNAs and their altered profile might be indicative of periodontitis. Here, we studied expression profiles of miRNAs in GCF and sought to illuminate their differences between healthy and periodontitis conditions. We could confirm differential expression patterns of selected 40 miRNAs in two GCF sample sets that were collected and analyzed independently. These results suggested that a subset of miRNAs are potentially useful as diagnostic biomarkers for periodontitis.

## Materials and methods

### Clinical subjects

Eight subjects (sample set #1; five healthy and three periodontitis; mean age: 38.0 and 52.0 years) contributed to the sampling of GCF used for comprehensive miRNA profiling (ready‐to‐use miRNA PCR panel for 752 miRNAs), and 12 subjects (sample set #2; six healthy and six periodontitis; mean age: 27.8 and 65.3 years) contributed to the sampling of GCF used for confirmation experiment (custom miRNA PCR panel for selected 40 miRNAs (Fig. 1). In total, 11 healthy and nine periodontitis subjects were studied. Diagnosis of periodontitis was primarily based on measurement of periodontal pocket depth (PD). Subjects having periodontal pockets with ≥ 4 mm PD were diagnosed as periodontitis. Clinical attachment level and percentage of bone loss were also recorded (Table 1). Aggressive periodontitis was distinguished from usual chronic periodontitis by detection of rapid progression of attachment loss and bone resorption for age in pocket and X‐ray examination. BOP was recorded after GCF sampling. All subjects were free of systemic diseases except one case of periodontitis complicated with mild diabetes without any medication. This study was approved by the Ethics Committee of the Faculty of Dentistry, Tokyo Medical and Dental University (TMDU; #1266). The periodontitis subjects were patients of the Department of Periodontics, Dental Hospital of TMDU, and the healthy subjects were volunteer dentists in the Department of Periodontology, TMDU. All individuals provided written informed consent to this study.

**Figure 1:** Study flowchart.

**Table 1:** Patient characteristics

	Sample		Age	Gender	Diagnosis	Treatment stage	Smoking	Full mouth			Sample sites			
								Mean PD (mm)	PD ≥ 4 mm sites (%)	BOP (%)	Mean PD (range; mm)	Mean CAL (range; mm)	BOP (%)	Bone loss (range; %)
Set #1	H	1	53	M	H		NS	1.8	0	0.0	2.0 (2)	2.0 (2)	−	
		2	43	M	H		NS	1.8	0	2.1	2.2 (2–3)	2.2 (2–3)	−	
		3	26	F	H		NS	1.8	0	3.6	2.4 (2–3)	2.4 (2–3)	−	
		4	37	F	H		S	1.8	1.4	3.5	1.8 (1–2)	1.8 (1–2)	−	
		5	31	M	H		NS	1.8	0.5	2.6	2.0 (2–3)	2.1 (2–4)	−	
	P	1	45	F	CP	During OHI	NS	2.8	21.6	29.6	4.8 (3–6)	6.0 (5–8)	+	47.7 (18.3–59.1)
		2	70	F	CP	After SRP	NS	2.7	12.5	5.6	6.7 (5–8)	8.0 (6–10)	+/−	66.6 (59.3–78.5)
		3	41	M	AgP	During OHI	S	3.6	32.7	51.8	6.3 (5–7)	7.5 (6–9)	+	63.6 (42.4–73.4)
Set #2	H	6	27	M	H		NS	2.0	0	1.8	2.6 (2−3)	2.6 (2−3)	–	
		7	27	M	H		NS	1.9	0	3.0	2.4 (2−3)	2.4 (2−3)	−	
		8	27	F	H		NS	2.2	0.6	3.6	2.0 (2)	2.0 (2)	−	
		9	30	F	H		NS	2.2	0	3.0	2.4 (2−3)	2.4 (2−3)	−	
		10	28	M	H		NS	2.3	1.2	2.4	2.6 (2−3)	2.6 (2−3)	−	
		11	28	F	H		NS	1.9	0	3.6	2.2 (2−3)	2.2 (2−3)	−	
	P	4	67	F	CP	After SRP	NS	2.5	15.8	14.2	4.8 (4–6)	5.6 (4–7)	+	56.2 (40.6–68.2)
		5	34	F	AgP	After SRP	NS	3.1	25.9	47.7	6.0 (4–8)	6.0 (4–8)	+	51.8 (29.5–64.1)
		6	73	M	CP	First visit	NS	4.4	75.7	94.4	6.2 (5−8)	6.2 (5−8)	+	42.6 (32.5–53.1)
		7	82	F	CP	After SRP	NS	2.3	9.4	13.0	5.0 (4−7)	6.7 (5–9)	+/−	81.7 (75.7–89.7)
		8	68	F	CP	After SRP	NS	3.1	35.2	55.6	6.2 (4−8)	6.4 (4–8)	+	57.6 (42.5–69.9)
		9	68	M	CP	During OHI	NS	2.3	9.0	16.7	4.0 (4)	5.0 (5)	+	33.9 (33.9)

M, male; F, female; H, healthy; CP, chronic periodontitis; AgP, aggressive periodontitis; PD, periodontal pocket depth; CAL, clinical attachment level; OHI, oral hygiene instruction; SRP, scaling and root planning; NS, nonsmoker; S, smoker; Bone loss: the ratio of the distance between cemento‐enamel junction (CEJ) and the bone crest to the whole root length from CEJ to the root apex.

### GCF sampling

Prior to sampling, the supragingival plaque and saliva around teeth were removed using a cotton pellet, and the teeth were air‐dried and isolated with cotton rolls. GCF samples were collected by gently inserting paper strips (PerioPaper®; Oraflow Inc., New York NY, USA) into the periodontal pocket as described previously 15. Any strip visibly contaminated with blood was discarded. Multiple strips were used for collecting approximately 4.8 μL of GCF for each subject. Given that the volume of GCF fully absorbed by a single strip corresponds to 1.2 μL, the sample volume was estimated based on the absorption levels of collected strips. In order to obtain a sufficient amount of GCF, multiple paper strips collected from several tooth sites were needed. The strips were pooled in tubes containing 60 μL of phosphate buffer, snap frozen, and subsequently used for RNA isolation.

### RNA isolation

RNA was extracted from GCF using the Trizol LS reagent (Life Technologies, Carlsbad, CA, USA) 16. Frozen GCF samples were dissolved in 750 μL of Trizol LS reagent and total volume of each sample was adjusted to 1 mL with RNase‐free water. Subsequently, 0.2 mL of chloroform was added, and aqueous phase of the mixture was collected and mixed with isopropanol. After centrifugation, the pellet was dried, rinsed with 80% ethanol, and dissolved in 50 μL of nuclease‐free water. RNA purity and concentration were evaluated by spectrophotometry using NanoDrop (ThermoFisher Scientific, Fremont, CA, USA). A260/230 ratios ranged from 0.9 to 1.6 while A260/280 ratios ranged from 1.6 to 1.8 among the GCF samples used for miRNA profiling. Quality of total RNA was assessed by the eukaryotic total RNA nano assay on Agilent 2100 BioAnalyzer (Agilent Technologies, Santa Clara, CA, USA), and electropherograms of all samples showed clear peaks for small RNAs.

### Expression profiling of miRNAs

To determine miRNA expression profiles, we used miRCURY LNA™ Universal RT microRNA PCR System (Exiqon, Vedbæk, Denmark) 17. The miRNA annotation of mirbase version 20.0 was used. Single‐stranded cDNA was synthesized by reverse transcription of 8 μL of RNA, using universal cDNA Synthesis Kit II (Exiqon). Diluted cDNA was mixed with ExiLENT SYBR® Green master mix (Exiqon), and quantitative PCR was performed using Roche LightCycler® 480 Real‐Time PCR system (Roche, Basel, Switzerland). The amplification result that did not reach the standard level after 40 cycles of PCR was discarded. In the first experiment (sample set #1), we used the Ready‐to‐Use miRNA PCR panel (Exiqon) for comprehensive screening of 752 miRNAs, and in the next experiment (sample set #2), we used a custom miRNA PCR panel for the selected 40 miRNAs.

For the analysis of sample set #1, the results of different samples were normalized by the global mean normalization method that is the gold standard for miRNA profiling studies that screen many miRNAs per sample 18. The average quantitation cycle (Cq) value was calculated for each sample and subsequently subtracted from each individual Cq value for that sample. To confirm the results in sample set #1, 40 miRNAs were selected and measured in sample set #2, and the results were analyzed by the multiple reference normalization method. The most stably expressed miRNAs were determined as reference probes by the previously reported algorithm 19. The data of each sample were normalized so that the average Cq values of reference probes were the same among the samples. The reference probes that recognize hsa‐miR‐324‐5p, hsa‐miR‐29c‐5p, hsa‐miR‐107, hsa‐miR‐324‐3p, and hsa‐miR‐30d‐5p were used for normalization. The normalized values were presented as delta Cq (ΔCq). The results are deposited in the Gene Expression Omnibus database (GSE89081).

### Public data of miRNA profiling in blood and gingival tissue

Expression profiles of miRNA in blood (GSE61741) and gingival tissue (GSE54710) were analyzed using geo2r bioinformatics tool 20. geo2r software was used to identify differential gene expression, and differences were considered significant for *P* < 0.05 after Benjamini–Hochberg false discovery rate (FDR) adjustment test. Blood samples from 18 periodontitis and 94 healthy subjects were compared by febit Homo Sapiens mirbase 13.0 (GSE61741). Gingival tissue samples from 159 periodontitis‐affected and 41 healthy sites were compared by Agilent 031181 Unrestricted Human miRNA V16.0 Microarray (GSE54710).

### Statistics

For each miRNA, *t*‐test was applied on normalized Cq values, and *P*‐value was calculated. Correction for multiple testing was done by using the Benjamini–Hochberg procedure, and FDR *q*‐value was calculated.

## Results

### Expression of miRNAs in GCF

First, we collected GCF from five healthy individuals and three periodontitis patients (sample set #1; Fig. 1). The sites of GCF sampling in healthy subjects had PD ≤ 3 mm with BOP negative, and those in diseased subjects had PD ≥ 4 mm (4–8 mm, except for one site with 3 mm in one subject) with mostly BOP positive. The details of subject characteristics and clinical parameters are shown in Table 1.

Next, we extracted RNA from GCF using the Trizol LS reagent, and RNA purity and concentration were evaluated by spectrophotometry using NanoDrop. We further analyzed the distribution of RNA size in GCF. Electropherograms of these samples showed peaks for small RNAs, the size of which was < 200 nt (Fig. 2). These observations suggested that RNA isolation procedure was successful for collecting small RNAs, and miRNAs could be included in the fraction of small RNAs. We did not observe ribosomal RNA peaks in the electropherograms of cell‐free GCF samples, which indicated that these samples were not contaminated with RNA derived from the cellular fraction.

**Figure 2:** Electropherograms of healthy and periodontitis GCF samples. Representative electropherograms of RNA samples derived from GCF of healthy (left) and periodontitis (right) subjects. In both samples, peaks of small RNAs whose size was less than 200 nucleotide were observed. The peak of size marker at 25 nt is shown.

### Distinctive expression patterns of miRNAs in GCF of periodontitis

Next, we aimed to efficiently screen mature miRNAs in GCF samples. PCR‐based quantitation of miRNAs by the miRCURY platform has previously shown better sensitivity and linearity for the low miRNA concentration range, and was suggested for the studies of body fluid samples that contain low levels of miRNAs 21. Hence, we attempted to detect miRNAs in GCF samples by miRCURY LNA™ microRNA PCR system, in which the cDNA template was amplified using miRNA‐specific and LNA‐enhanced forward and reverse primers. This system successfully detected substantial amounts of mature miRNAs in GCF samples. Furthermore, the result of miRNA profiling in GCF revealed clear differences between healthy and periodontitis samples (Table S1). Two‐dimensional scatter plot of miRNA expression patterns of healthy and periodontitis GCF samples was illustrated by principal component analysis (PCA), which clearly distinguished between these two groups (Fig. 3A).

**Figure 3:** Expression profiling of miRNAs in GCF sample set #1. (A) PCA of miRNA expression profiles. Two‐dimensional scatter plot represents the differential miRNA expression patterns of healthy (H1–H5; *n* = 5) and periodontitis (P1–P3; *n* = 3) GCF samples (sample set #1). The *x*‐axis indicates PCA Component 1 (PC1: 46.9% variance) and the *y*‐axis shows PCA Component 2 (PC2: 15.7% variance). (B**)** Volcano plot showing differential expression of miRNAs between healthy and periodontitis subjects. The *x*‐axis represents relative expression ratios shown as −ΔΔCq values. The *y*‐axis indicates −log_10_(FDR *q*‐value) between the two groups. The lines indicate cutoff of FDR *q*‐value < 0.05 and |ΔΔCq| > 1.0. Red dots are miRNAs that meet these criteria.

This quantitative miRNA expression platform contained prealiquoted PCR primer sets for 752 human miRNAs, and we obtained expression data of 619 miRNAs in at least one sample of both healthy and periodontitis groups. Among them, 332 and 287 miRNAs were up‐ and down‐regulated in periodontitis, respectively (Fig. 3B). Setting the criteria of FDR *q*‐value < 0.05 and the difference of ΔCq value (ΔΔCq) > 1.0 or < −1.0, we identified 40 and 46 miRNAs that showed up‐ and down‐regulation in periodontitis GCF samples (Fig. 3B).

We compared these differentially expressed miRNAs in GCF to those previously identified in blood and gingival tissue samples of periodontitis 22. Up‐ and down‐regulated miRNA sets determined in different sample types were compared, and we noted that they are mostly distinctive (Fig. 4). Of particular note, hsa‐miR‐210‐3p was found to be commonly down‐regulated in three different sample types of periodontitis.

**Figure 4:** Differentially expressed miRNAs in GCF, blood, and gingival tissue samples. Comparisons of our result in GCF, and those obtained from GSE61741, and GSE54710 datasets.

Next, we performed pathway analysis using the list of 40 up‐regulated and 46 down‐regulated miRNAs in periodontitis GCF samples. We applied diana‐mirpath v3.0, an online software, for the functional annotation of miRNAs, and performed KEGG pathway‐enrichment analysis based on the DIANA‐microT‐CDS miRNA target prediction algorithms 23. Interestingly, miRNAs up‐regulated in periodontitis were related to transforming growth factor‐β (TGF‐β) signaling while down‐regulated miRNAs were associated with ErbB signaling (Fig. 5). These results suggested that altered expression of miRNAs in GCF of periodontitis might have functional impact on molecular signals in the gingival tissues.

**Figure 5:** Pathway analysis. KEGG pathway analysis of the 40 up‐regulated (−ΔΔCq > 1.0, FDR < 0.05) and 46 down‐regulated (−ΔΔCq < −1.0, FDR < 0.05) miRNAs in periodontitis that were identified in GCF sample set #1. The predicted pathways are presented in the order of −log_10_(*P*‐value).

### Selection of 40 miRNAs differentially expressed in GCF of periodontitis

Based on the result of miRNA profiling in GCF samples, we selected 40 miRNAs for further confirmation experiments in GCF samples obtained from different subjects (sample set #2; Fig. 1). The sites of GCF sampling in healthy subjects had PD ≤ 3 mm with BOP negative, and those in diseased subjects had PD ≥ 4 mm (4–8 mm) with mostly BOP positive (Table 1).

We compared our miRNA profiling result with the lists of differentially expressed miRNAs in periodontitis gingival tissues that have been described in three previous reports 22, 24, 25. Finally, we selected 40 miRNAs whose differential expression is preferably observed both in GCF and gingival tissues. Among them, 19 and 21 miRNAs were up‐ and down‐regulated, respectively, in periodontitis GCF samples (sample set #1).

To determine the optimal miRNAs for normalization whose expression levels were stable among all samples, we employed a previously reported algorithm 19. Candidate miRNAs were ranked according to their expression stability, and we selected hsa‐miR‐324‐5p, hsa‐miR‐29c‐5p, hsa‐miR‐107, hsa‐miR‐324‐3p, and hsa‐miR‐30d‐5p as reference miRNAs. Thus, the measurement of these miRNAs was included in the following experiments as reference probes for the normalization of miRNA levels in GCF samples.

### Distinctive expression patterns of 40 miRNAs in GCF of periodontitis

To confirm the results in sample set #1, we measured the expression levels of selected 40 miRNAs in GCF from sample set #2 (Table S2). The sites of GCF sampling in healthy subjects had PD ≤ 3 mm with BOP negative, and those in diseased subjects had PD ≥ 4 mm (4–8 mm) with mostly BOP positive. The details of subject characteristics and clinical parameters are shown in Table 1. The results showed differences between six healthy and six periodontitis subjects, and the heatmap displayed clear contrast (Fig. 6A). The expression levels of 33 miRNAs showed significant differences with FDR *q*‐value < 0.05, and 17 miRNAs displayed ΔΔCq > 1.0 or < −1.0 (Fig. 6B). Judging from the ΔCq values, relatively high expression levels of hsa‐miR‐223‐3p, hsa‐miR‐203a and hsa‐miR‐205‐5p in GCF samples of periodontitis patients were confirmed (Fig. 6C).

**Figure 6:** Expression of selected 40 miRNAs in GCF sample set #2. (A) Two‐dimensional hierarchical clustering of miRNA expression levels in healthy (H6‐H11; *n* = 6) and periodontitis (P4‐P9; *n* = 6) GCF samples (sample set #2). Red to blue color gradient of heatmap shows the relative expression levels based on −ΔCq values. The results of 40 selected miRNAs except hsa‐miR‐20a‐5p are displayed since amplification for hsa‐miR‐20a‐5p failed in the P7 sample. (B) Volcano plot showing differential expression of miRNAs between healthy and periodontitis subjects. The *x*‐axis represents relative expression ratios shown as −ΔΔCq values. The *y*‐axis indicates −log_10_(FDR *q*‐value) between the two groups. The lines indicate cut‐off of FDR *q*‐value < 0.05 and |ΔΔCq| > 1.0. Red dots are miRNAs that meet these criteria. (C) Box plot showing expression levels of miRNAs indicated as −ΔCq. Red and green boxes represent the values of healthy (*n* = 6) and periodontitis (*n* = 6) groups, respectively. The central line in the box indicates the median value. The result of hsa‐miR‐20a‐5p expression in the periodontitis group was obtained from five samples. The upper panel shows the values of 19 up‐regulated miRNAs while the lower panel shows the values of 21 down‐regulated miRNAs.

Next, we selected pairs of healthy and periodontitis subjects so that age and gender match, and compared the expression levels of the 40 miRNAs, that is, H2 vs. P3 (sample set #1), H4 vs. P1 (sample set #1), and H9 vs. P5 (sample set #2). As observed in the overall comparison of sample set #2 (Fig. 6A), the selected 40 miRNAs exhibited similar up‐ and down‐regulation patterns in these three different pairs (Fig. 7).

**Figure 7:** Comparison of the age‐ and gender‐matched pairs. Expression levels of 40 selected miRNAs in three age‐ and gender‐matched pairs of healthy and periodontitis subjects. H2 vs. P3 (sample set #1), H4 vs. P1 (sample set #1), and H9 vs. P5 (sample set #2). Note that up‐ and down‐regulation patterns are mostly common among three comparison pairs.

Furthermore, up‐ and down‐regulation pattern of each miRNA was compared between sample set #1 (five healthy and three periodontitis) and sample set #2 (six healthy and six periodontitis). Surprisingly, all of 40 miRNAs showed the same patterns, and 19 miRNAs were up‐regulated while 21 miRNAs were down‐regulated in periodontitis GCF of both sample sets. When the ΔΔCq values of these miRNAs between sample set #1 and sample set #2 were compared, high correlation was observed (Fig. 8A). Finally, we compared the distribution of ΔCq values of the 19 up‐regulated and 21 down‐regulated miRNAs among the GCF samples used in this study, and observed distinctive expression patterns in both sample sets (Fig. 8B). These reproducible results implied that the selected 40 miRNAs are potentially useful biomarkers for periodontitis.

**Figure 8:** Comparison of the results from two different sample sets. (A) Scatter plot showing correlation of the 40 miRNA expression ratios (−ΔΔCq values) obtained from two different sample sets. Each dot represents the −ΔΔCq value of each miRNA that was obtained by comparison between healthy and periodontitis groups in sample set #1 (*y*‐axis) and sample set #2 (*x*‐axis). Spearman's correlation coefficient (ρ) = 0.95. (B) Box plot showing expression levels of 40 miRNAs indicated as −ΔCq. Red and green boxes represent the values of healthy and periodontitis samples, respectively. The results of different sample sets are presented separately. The upper panel shows the values of 19 up‐regulated miRNAs while the lower panel shows the values of 21 down‐regulated miRNAs. The central line in the box indicates the median, lower box bound the first quartile, and upper box bound the third quartile.

## Discussion

This study is the first to verify the presence of miRNAs in GCF. We further discovered that GCF from periodontitis patients has unique miRNA profiles. Several studies have proved that expression patterns of miRNAs in gingival tissues could be used to distinguish periodontitis patients from healthy subjects 22, 24, 25. Our finding suggests that miRNA detection in GCF may serve as a novel diagnostic tool that circumvents the invasive procedure to obtain biopsy samples of gingival tissues.

Due to the small size and low abundance of mature miRNAs, their detection in body fluids has been technically hampered. However, in recent years, several methods have been developed, including small RNA sequencing, microarray hybridization, and quantitative RT‐PCR. A recent study has systematically compared the performance of these different platforms, and demonstrated that quantitative RT‐PCR method is highly sensitive, specific, and thus superior to the other methods, especially for low input RNA samples 26. Hence, we applied this system to GCF samples to obtain reliable quantitation of miRNAs, and successfully detected miRNAs in GCF, for the first time.

By using the ready‐to‐use miRNA PCR panel for comprehensive profiling, we could detect 619 miRNAs in GCF samples, and setting the criteria of FDR *q*‐value < 0.05, and ΔΔCq > 1.0 or < −1.0, we identified 40 up‐regulated and 46 down‐regulated miRNAs in GCF of periodontitis. We further selected 40 miRNAs for the custom PCR panel, and confirmed their differential expression between control and periodontitis in an independently collected GCF sample set. Comparative analyses on the results of different sample sets demonstrated that up‐ and down‐regulation patterns of these miRNAs were reproducible. It should be noted that we also defined reference miRNAs suitable for the normalization of miRNA expression levels in GCF samples.

In a previous report on gingival tissues with a relatively large sample size, four miRNAs (hsa‐miR‐451, hsa‐miR‐223, hsa‐miR‐486‐5p, and hsa‐miR‐3917) and seven miRNAs (hsa‐miR‐1246, hsa‐miR‐1260, hsa‐miR‐141, hsa‐miR‐1260b, hsa‐miR‐203, hsa‐miR‐210, and hsa‐miR‐205*) were identified to be overexpressed and underexpressed in periodontitis (*n* = 158) compared to controls (*n* = 40), respectively 22. In agreement with these previous observations, hsa‐miR‐451a, hsa‐miR‐223‐3p, hsa‐miR‐486‐5p, hsa‐miR‐1260a, hsa‐miR‐203a, hsa‐miR‐210‐3p, and hsa‐miR‐205‐3p showed similar up‐ and down‐regulation patterns in periodontitis GCF samples of the present study. As such, it is conceivable that periodontitis‐associated miRNAs are largely common between gingival tissues and GCF samples.

A hallmark of periodontitis is disorganized extracellular matrix (ECM) in the gingival tissues, and fibroblast plays a central role to regulate ECM turnover and remodeling. Thus, gingival fibroblasts are essential not only for the homeostasis of gingival tissue architecture but also for the pathogenesis of periodontitis. Most recently it has been reported that hsa‐miR‐223 positively regulates the expression of IL‐1β and IL‐6 in human gingival fibroblasts 27. In the present study, we noticed that hsa‐miR‐223‐3p was the most highly expressed miRNA in GCF samples and was up‐regulated in periodontitis. Taken together, hsa‐miR‐223‐3p might represent a promising GCF biomarker which reflects the inflammatory status of gingival tissues.

We have recently identified that vascular endothelial growth factor (VEGF) signal mediated by VEGF receptor 1 (VEGFR1: also known as FLT1) is crucial for the phenotype of periodontitis‐associated fibroblasts to potentially promote the progression of periodontitis 28. Intriguingly, a subset of selected 40 miRNAs has been demonstrated to target VEGF‐A or FLT1, including hsa‐miR‐200b‐3p, hsa‐miR‐200c‐3p, hsa‐miR‐203a‐3p, and hsa‐miR‐205‐5p 29. These miRNAs were down‐regulated in periodontitis GCF samples, which might be associated with enhanced VEGF signaling in periodontitis‐associated fibroblasts.

The members of miR‐200 family and miR‐205 are involved in specification of the epithelial phenotype and are negatively regulated by TGF‐β 30. We found that most miRNAs of the miR‐200 family (miR‐200a, miR‐200b, and miR‐200c) and miR‐205 were down‐regulated in periodontitis GCF samples. This finding was in accordance with our previous report that TGF‐β signaling is activated in periodontitis 31. Collectively, suppression of these miRNAs might be a result of enhanced TGF‐β signaling in periodontitis and linked to dysregulated gingival epithelial regeneration in the pathogenesis of periodontitis.

A limitation of the current study was the small sample size. Further studies using large cohorts are necessary. Despite this limitation, it was noteworthy that the differential expression patterns (up‐ or down‐regulation) of selected 40 miRNAs yielded very similar results between two different sample sets. We could also confirm similar patterns among age‐ and gender‐matched comparisons between healthy and periodontitis subjects (Fig. 7). As another limitation, we included patients of both chronic and aggressive periodontitis that are known to have different clinical, microbial, and immunological characteristics. It should be noted that the main purpose of this study was to detect a differential profile between periodontitis and health conditions, but not regarding the activity or subtype of periodontitis.

In summary, we showed that GCF of periodontitis displays a unique profile of miRNAs compared to that of the healthy control. Our study suggests that miRNA detection in GCF holds potential as a diagnostic tool for periodontitis. Profiling of miRNAs in GCF samples might provide quantitative, objective, and even mechanistic information that improves the management of periodontitis.

## Author contributions

AA, YY, YI, and MO were involved in conceptualization, funding acquisition, and supervision. KE, AA, SK, SM, SS, SK, and YI contributed toward methodology, resources, investigation, validation, formal analysis, and project administration. MH was involved in software and visualization. AS, MH, YY, TY, and MO were involved in data curation. AS, MH, YY, AA, YI, and MO were involved with writing.

## Supporting information


**Table S1.** Expression profiling of miRNAs in GCF sample set #1.

**Table S2.** Expression of selected 40 miRNAs in GCF sample set #2.
